The article "Research and Application of Clustering Algorithm for Text Big Data" was published in 2022. Journal: Comput Intell Neurosci.

# Research and Application of Clustering Algorithm for Text Big Data

**DOI:** 10.1155/2022/7042778

**Published:** 2022-06-08

**Authors:** Zi Li Chen

**Affiliations:** Institute of General Aviation Industry, Fujian Chuanzheng Communications College, Fuzhou 350007, China

## Abstract

In the era of big data, text as an information reserve database is very important, in all walks of life. From humanities research to government decision-making, from precision medicine to quantitative finance, from customer management to marketing, massive text, as one of the most important information carriers, plays an important role everywhere. The text data generated in these practical problems of humanities research, financial industry, marketing, and other fields often has obvious domain characteristics, often containing the professional vocabulary and unique language patterns in these fields and often accompanied by a variety of “noise.” Dealing with such texts is a great challenge for the current technical conditions, especially for Chinese texts. A clustering algorithm provides a better solution for text big data information processing. Clustering algorithm is the main body of cluster analysis, K-means algorithm with its implementation principle is simple, low time complexity is widely used in the field of cluster analysis, but its *K* value needs to be preset, initial clustering center random selection into local optimal solution, other clustering algorithm, such as mean drift clustering, K-means clustering in mining text big data. In view of the problems of the above algorithm, this paper first extracts and analyzes the text big data and then does experiments with the clustering algorithm. Experimental conclusion: by analyzing large-scale text data limited to large-scale and simple data set, the traditional K-means algorithm has low efficiency and reduced accuracy, and the K-means algorithm is susceptible to the influence of initial center and abnormal data. According to the above problems, the K-means cluster analysis algorithm for data sets with large data volumes is analyzed and improved to improve its execution efficiency and accuracy on data sets with large data volume set. Mean shift clustering can be regarded as making many random centers move towards the direction of maximum density gradually, that is, moving their mean centroid continuously according to the probability density of data and finally obtaining multiple maximum density centers. It can also be said that mean shift clustering is a kernel density estimation algorithm.

## 1. Introduction

Text detection is the fundamental step in many computer vision applications. This paper introduces a novel text detection technique, and we verify the utility of the method in the YouTube video text dataset and find that the method runs more than 2 times [1] of the classical method. This paper expounds the existing research work on the decomposition and inference of clustering algorithms based on text big data and points out the shortcomings of the existing research work [2]. Big data text analysis is the promoter of knowledge management. This paper believes that, through the big data text analysis, it not only can improve the quality of life of ordinary people but also can make various enterprises for benign competition, so as to improve the quality of enterprises. This paper provides many different opinions, involving many aspects, from the daily life of ordinary people to different business functions of enterprises, from stock market to finance. Text big data analysis has become a shortcut and a leader of knowledge management [3]. Big data is used in various industries, which contains various value information, and text big data, as an important part of big data, carries countless human knowledge. This paper reviews the feature representation of text big data and finally discusses the future trend of large-text data content understanding [4]. Nowadays, the application of big data is not open in various fields, and the meaningful analysis and extraction of big data are needed in many fields. In this paper, we study the cluster analysis process based on text big data and propose the whole process [5] from collecting big data to applying various clustering algorithms for cluster analysis. This paper uses K-means text clustering algorithm to analyze the big data talent recruitment information. The results show that big data jobs are concentrated in frontier cities. Most enterprises require undergraduate or graduate students, and a few enterprises see whether the applicant has many years of relevant work experience. There are wage differences between different types of jobs, and the higher the position, the higher the requirements for education and experience will be [6]. Discovering knowledge from text data in a high-speed and accurate manner is a major challenge in large-text data mining. This paper presents a new large-text data mining method, the random walk algorithm, which accurately extracts two basic and complementary words from numerous text data. We show that the proposed random walk algorithm is based on the aggregate relation and the combined relation [7] in recent decades, with the development of the Internet, it is almost normal for people to use mobile phones and computers, while the phenomenon of reading books decreases day and night. This also makes the storage and search of articles in the digital library reach an unprecedented height, but it is limited to indexing the text description of each pseudocode and cannot provide simple algorithm-specific information. Therefore, this paper proposes a set of algorithms to extract and search related information from text big data, and its efficiency is as high as 78% through practical verification [8] accurate. The K-means algorithm is an incremental clustering method. In this paper, we propose improvements of the algorithm to reduce the computational amount without significantly affecting the quality of the solution. It is also tested and showed that the improved K-means algorithm has better results than [9]. This paper presents a new algorithmic model, called the fuzzy c-mean clustering model (or FCM). FCM solves the problem [10] that objects in the dataset cannot partition significantly separated clusters. We discuss three main issues of traditional partitioning clustering, namely, sensitivity to initialization, difficulty determining the number of clusters, and sensitivity [11] to noise and outliers. In this paper, we propose an adaptive spatial fuzzy C mean clustering algorithm for the segmentation of 3D MR images in text big data. We verify the effectiveness of [12] through extensive segmentation experiments on simulation and real MR images and comparison with existing algorithms. Clustering algorithm plays an important role in analyzing the structure and function of biological network. In this paper, a fast local network clustering algorithm SPICI is proposed. It has the most advanced performance and can cluster all the test networks in a very short time. Experiments show that its success rate is the highest among other algorithms. Reference [13] in terms of the quality of the clusters it finds. In the data analysis methods, we often use the cluster analysis. In this paper, we propose K-means clustering algorithms and investigate the problem where the K-means clustering algorithm is limited to small-scale datasets. Finally, this paper presents a method to make the algorithm more efficient and thus obtain better clustering [14] with reduced complexity. In text big data processing, K-means is our common partitioning clustering algorithm. However, the proposed algorithm is still unsatisfied in some professional fields, and many initialization methods have been proposed to solve this problem. In this paper, we demonstrate that popular initialization methods generally perform poorly, and that there are actually some powerful alternatives to these methods [15].

The article "Research and Application of Clustering Algorithm for Text Big Data" was published in 2022. Journal: Comput Intell Neurosci.

## 2. Text Big Data and Cluster Analysis

### 2.1. Text Big Data

Text big data refers to the document data, which is manifested in the form of documents and contains a large amount of information, fast speed, more types, and low data value. In big data, text big data is an important part of big data. Due to the rapid development of information technology, the growth rate of data sources increases through the media of mobile phones and computers. Text big data has three characteristics: diversity, large quantity, and fast speed. For the data collection technology, there are still huge challenges to ensure its accuracy and effectiveness.

### 2.2. Mining and Application of Big Data

Data mining refers to a process of searching for the information hidden in the data through algorithms, which is the process of analyzing the hidden and potentially valuable information contained in a large amount of data in a database. Data mining does not need manual operation, can automatically analyze the data of enterprises, can summarize the data, and then make reasoning, to help decision makers to adjust market strategies, reduce risks, and make correct decisions. The practical data analysis of big data can help people make judgments so as to take appropriate actions. Because of the popularity of the network and the convenience of big data application, the application of big data is more and more extensive such as answering customer questions, meeting customer service needs, helping to optimize business processes, improving health care and research and development, and so on. With the continuous innovation of big data in various industries, big data will gradually create more value for human beings. Text clustering is to cluster some documents with similar contents from many documents. Simply speaking, it is to find any two most relevant text information in the text information space and degenerate them into one text information, so as to reduce the amount of information.

### 2.3. Text Big Data Processing Method

Nowadays, our common text big data processing method is cluster analysis, which is a quantitative method. When processing text big data, clustering score is generally analyzed from two perspectives. First, from the perspective of data analysis, it is a multivariate statistical analysis method for quantitative analysis of multiple samples. Second, from the perspective of data mining, it can be divided into division clustering, hierarchical clustering, density-based clustering, and network-based clustering. Partition clustering is based on distance clustering, which effectively uses mean or center point and small data. Hierarchical clustering is a very intuitive algorithm, as its name implies, it is to cluster layer by layer. Density-based clustering is to divide data into each category according to the connection of density around it. Grid-based clustering adopts multiresolution grid data structure, which can process data quickly.

The article "Research and Application of Clustering Algorithm for Text Big Data" was published in 2022. Journal: Comput Intell Neurosci.

### 2.4. Type of Clustering Algorithm

#### 2.4.1. Cluster Analysis

Clustering is a technology of classifying data by computer, is also a classification of multivariate statistical analysis method, divides a data set according to a specific standard into different classes or clusters, and makes the similarity of the data object as big as possible, not the difference in the same cluster is as big as possible. Text clustering refers to the clustering of documents. Similarly, data with similar characteristics are gathered together as much as possible, and dissimilar data are separated as far as possible. Not only text can be clustered, but anything where features can be extracted. For example, e-commerce websites cluster goods according to features such as price and color, app stores according to the App's user age and downloads, and movie websites according to the theme and year of films. Machine learning including clustering can be performed simply by converting real-life objects into a vector in the mathematical world through feature extraction.

#### 2.4.2. Clustering Algorithm

When dealing with text big data, we all have an algorithm bias, and we use different algorithms to deal with different problems. The following clustering algorithms are commonly used when we cluster data.

## 3. Cluster Algorithm Analysis

### 3.1. Definition of the Class

**Definition 1 .**

Set the positive number given by the threshold *T*, if the distance *d* of any two elements in the set *G*_*ij*_. Everything meets

(1) $$\begin{array}{c} d_{ij}\leq T,\;\left(i,j\in G\right). \end{array}$$

It is called that *G* constitutes a class for the threshold *T*.

**Definition 2 .**

Let the threshold *T* be the given positive number, if each *i* ∈ *G* in the set *G* satisfies

(2) $$\begin{array}{c} \frac{1}{n-1}\sum_{j\in G}d_{ij}\leq T\underset{x⟶\infty }{\lim}, \end{array}$$

where *n* is the number of elements in the set *G* and then *G* is said to form a class for the threshold *T*.

**Definition 3 .**

Let *T* and *H* (*H* > *T*) be two given positive numbers, if the average pairwise element distance in the set *G* meets

(3) $$\begin{array}{c} \frac{1}{n\left(n-1\right)}\sum_{i\in G}\sum_{j\in }d_{ij}\leq T,\;d_{ij}\leq H\left(i,j\in G\right), \end{array}$$

where *n* is the number of elements in the set *G* and *G* is called a class of *H* for the threshold *T*.

Formula (2) shows that the average of the sum of distances between any two elements in the set *G* is less than a given threshold *T*. Similarly, formula (3) indicates that the average is less than *T* and less than *H*.

The article "Research and Application of Clustering Algorithm for Text Big Data" was published in 2022. Journal: Comput Intell Neurosci.

### 3.2. Characteristics of the Class

Let the sample contained by class *G* be *X*_(1)_, *X*_(2)_,…, *X*_(*N*)_, where *t* is the sample of population *G* and its characteristics can be characterized from different angles. The barycenter of *G*, sample deviation matrix *A*_G_, and sample covariance matrix *S*_G_ and *D*_G_ represent the diameter of class *G* as follows:

(4) $$\begin{array}{c} {\bar{X}}_{G}=\frac{1}{n}\sum_{t=1}^{n}X_{\left(t\right)}, \end{array}$$

(5) $$\begin{array}{c} A_{G}=\sum_{T=1}^{n}\left(X_{\left(\text{t}\right)}-{\bar{X}}_{G}\right), \end{array}$$

(6) $$\begin{array}{c} D_{G}=\sum_{t-1}^{n}\left(X_{\left(t\right)}-{\bar{X}}_{G}\right),\\ \left(X_{\left(t\right)}-{\bar{X}}_{G}\right)=\text{tr}\left(A_{G}\right), \end{array}$$

(7) $$\begin{array}{c} D_{G}=\underset{i,j\in G}{\max}d_{i,j}. \end{array}$$

### 3.3. Distance

If *n* samples are considered as *n* points in m-dimensional space, then the similarity between two samples is *d*_*i*,*j*_ measure. For sample *X*_*i*_, the distance of *X*_*j*_, the general requirement is *d*_*ij*_ ≥ 0, for any *i*, *j*, when *d*_*ij*_=0⇔*X*_(*i*)_=*X*_(*j*)_; *d*_*ij*_=*d*_*ji*_, for any *i*, *j*; *d*_*ij*_ ≤ *d*_*ik*_+*d*_*kj*_, for any *i*, *j*, *k* (triangle inequality).

The common distances are as follows.

The Minkowski distance is represented as

(8) $$\begin{array}{c} d_{ij}\left(q\right)={\left[{\sum_{t=1}^{m}\left|x_{it}-x_{jt}\right|}^{q}\right]}^{1/q},\;\left(i,j=1,2,\ldots ,n\right). \end{array}$$

The first order Ming distance at *V* is expressed as

(9) $$\begin{array}{c} d_{ij}\left(1\right)=\sum_{t=1}^{m}\left|x_{it}-x_{jt}\right|,\;\left(i,j=1,2,\ldots ,n\right). \end{array}$$

The absolute distance, when *X*, is expressed as

(10) $$\begin{array}{c} d_{ij}\left(2\right)={\left[\sum_{t=1}^{m}{\left|x_{it}-x_{jt}\right|}^{2}\right]}^{1/2},\;\left(i,j=1,2,\ldots ,n\right). \end{array}$$

Euclidean distance, when to *Z*, is represented as

(11) $$\begin{array}{c} d_{ij}\left(\infty \right)=\underset{1\leq t\leq m}{\max}\left|x_{it}-x_{jt}\right|\;\left(i,j=1,2,\ldots ,n\right). \end{array}$$

That is, the Chebyshev distance.

The Mahalanobis distance is located.

In 1930s, Mahala Mahalanobis, a famous Indian mathematician, put forward Mahalanobis distance, which is of great significance in data clustering. Σ is the covariance array of the indicator, ∑=(*ω*_*ij*_)_*p*×*p*_, as shown in (12) and (13) among

(12) $$\begin{array}{c} \omega_{ij}=\frac{1}{n-1}\sum_{\alpha =1}^{n}\left(x_{\alpha i}-{\bar{x}}_{i}\right)\left(x_{\alpha j}-{\bar{x}}_{j}\right),\;i,j=1,2,\ldots ,p, \end{array}$$

(13) $$\begin{array}{c} {\bar{x}}_{i}=\frac{1}{n}\sum_{\alpha =1}^{n}x_{\alpha i}, \end{array}$$

When ∑^−1^ is present, it is Ma distance, which can be expressed as

(14) $$\begin{array}{c} d_{ij}^{2}\left(M\right)={\left(X_{i}-X_{j}\right)}^{'}\sum^{-1}\left(X_{i}-X_{j}\right). \end{array}$$

The Mahalanobis distance from sample *X* factory to population *G* port is defined as

(15) $$\begin{array}{c} d^{2}\left(X,G\right)={\left(X-\mu \right)}^{'}\sum^{-1}\left(X-\mu \right). \end{array}$$

Here, *μ* is the mean vector of the population.

The article "Research and Application of Clustering Algorithm for Text Big Data" was published in 2022. Journal: Comput Intell Neurosci.

The Lance and Williams Distance, also known as the Canberra Distance, is considered a weighted version of the Manhattan distance.

The Rand distance is a kind of distance given by Lance and Williams. The formula is calculated as follows:

(16) $$\begin{array}{c} d_{ij}\left(L\right)=\frac{1}{m}\sum_{t=1}^{m}\frac{\left|x_{it}-x_{jt}\right|}{x_{it}+x_{jt}}, \end{array}$$

(17) $$\begin{array}{c} d_{ij}\left(L\right)=\frac{1}{m}\sum_{t=1}^{m}\frac{\left|x_{it}-x_{jt}\right|}{x_{it}+x_{jt}},\;i,j=1,2,\ldots ,n. \end{array}$$

Jeffery and Matasta put forward the distance formula, but there is no related reference. The formula is calculated as

(18) $$\begin{array}{c} d_{ij}\left(J\right)={\left[\sum_{k=2}^{p}{\left(\sqrt{x_{ik}-x_{jk}}\right)}^{2}\right]}^{1/2}. \end{array}$$

Incline intersection space distance is defined as follows.

Since there are often different correlations between the variables, the distance of the orthogonal space calculates the sample space as variable.

You can use the oblique intersection space distance. The calculation formula is

(19) $$\begin{array}{c} d_{ij}={\left[\frac{1}{p^{2}}\sum_{n=1}^{p}\sum_{k=1}^{p}\left(x_{ih}-x_{jh}\right)\left(x_{ik}-x_{jk}\right)r_{hk}\right]}^{1/2}. \end{array}$$

### 3.4. Similarity Coefficient

To study the relationship between the samples, the similarity coefficient method was used here. First, the samples are classified, and then the relationship between the samples is studied by the similarity coefficient. *C*_*ij*_ represents the similarity coefficient between samples *X*_*i*_ and *X*_*j*_, with *C*_*ij*_=±1⇔*X*_*i*_=*aX*_*j*_; |*C*_*ij*_| ≤ 1, valid for any *i*, *j*; *C*_*ij*_=*C*_*ji*_ is true for any *i*, *j*. The closer the absolute value of *C*_*ij*_ is to 1 here, the more similar them *X*_*i*_ and *X*_*j*_ are. Conversely, the two are estranged. The common similarity coefficients are angular cosine:

(20) $$\begin{array}{c} c_{ij}\left(1\right)=\cos\;\alpha_{ij}\frac{\sum_{k=1}^{n}x_{ki}x_{kj}}{{\left[\left(\sum_{k=1}^{n}x_{ki}^{2}\right)\left(\sum_{k=1}^{n}x_{kj}^{2}\right)\right]}^{1/2}}. \end{array}$$

When *X*_*i*_ and *X*_*j*_ are parallel, the angles *α*_*ij*_=0^0^ and *C*_*ij*_(1)=1 indicate that the two vectors are completely similar; when *X*_*i*_ and *X*_*j*_ are orthogonal, the angles *α*_*ij*_=90^0^ and *C*_*ij*_(1)=0 indicate that the two vectors are not correlated.

The article "Research and Application of Clustering Algorithm for Text Big Data" was published in 2022. Journal: Comput Intell Neurosci.

The correlation coefficient is expressed as

(21) $$\begin{array}{c} c_{ij}\left(2\right)=\cos\;\alpha_{ij}\frac{\sum_{k=1}^{n}\left(x_{ki}-{\bar{x}}_{i}\right)\left(x_{kj}-{\bar{x}}_{j}\right)}{{\left\{\left[\sum_{k=1}^{n}{\left(x_{ki}-{\bar{x}}_{i}\right)}^{2}\right]\left[\sum_{k=1}^{n}{\left(x_{kj}-{\bar{x}}_{j}\right)}^{2}\right]\right\}}^{1/2}}. \end{array}$$

I indicates the linear correlation of the two vectors.

### 3.5. K-Means Clustering Algorithm

The original mean clustering algorithm is different from the improved mean clustering algorithm. The specific steps of the original clustering algorithm are as follows: input data set *X*={*x*_1_, *x*_2_,…*x*_*n*_}, cluster number K; output K cluster *C*_*j*_, *j*=1,2,…., *k*, make *I*=1, and randomly select K data points as the initial cluster center *m*_*j*_(*I*), *j*=1,2,…, *k*. Of K clusters; calculate the distance between each data point and the center of the K cluster *d*(*x*_*i*,_*m*_*j*_(*I*)), *i*=1,2,…., *n*, *j*=1,2,…., *k*, if it meets

(22) $$\begin{array}{c} d\left(x_{i,}m_{j}\left(I\right)\right)=\min\left\{d\left(x_{i},m_{j}\left(I\right)\right),\;j=1,2,\ldots ,k\right\}. \end{array}$$

Then, calculating *S* new clustering centers satisfies

(23) $$\begin{array}{c} m_{i}\left(I+1\right)=\frac{1}{N_{j}}\sum_{i=1,x_{i}\in C_{j}}^{N_{j}}x_{i},\;j=1,2,\ldots ,k. \end{array}$$

If *m*_*j*_(*I*+1) ≠ *m*_*j*_(*I*), *j*=1,2,…., *k*, then *I*=*I*+1, return to step 2. Otherwise, the algorithm ends.

K-means clustering algorithm can also add clustering criterion function to terminate the iterative process; generally, the criterion function of sum of squares of clustering errors is adopted, that is, the sum of squares of clustering errors *J* is calculated in the fourth step of the above algorithm flow, and then judgment is added. If the value of *J* does not change obviously twice, it means that the value of *J* has converged, and the algorithm is ended. Otherwise, it is transferred to the second step to continue execution. Specifically, *K* clustering centers (*m*_1_,*m*_2_,…,*m*_*k*_) are randomly designated as follows. Assign *x*_*i*_, for any *x*_*i*_, the nearest to it is divided into the same class. Recalculate the center of each cluster with formula *H*

(24) $$\begin{array}{c} m_{i}\frac{1}{N_{i}}\sum_{j=1}^{N_{i}}x_{ij},\;i=1,2,\ldots ,n. \end{array}$$

The deviation is then calculated using formula *F*

(25) $$\begin{array}{c} J={\sum_{i=1}^{k}\sum_{j=1}^{n_{i}}\left\|x_{ij}-m\right\|}^{2}. \end{array}$$

If *J* converges, the returm(*m*_1_, *m*_2_,…, *m*_*k*_) algorithm ends; otherwise, proceed to the second step.

The article "Research and Application of Clustering Algorithm for Text Big Data" was published in 2022. Journal: Comput Intell Neurosci.

The idea of the original clustering algorithm is reflected in the above algorithm process, from which we can see that the selection of the initial cluster center point of each cluster is crucial to the final result of the clustering. In the above algorithm, the focus is on the iterative algorithm. In each iteration of the formula, the data points are divided into the cluster with the nearest cluster center and then recalculate the cluster center and then repeatedly iterate until each data point is no longer redivided. Simply put, K-means is a method of dividing data into K parts without any supervision signal.

## 4. Study on Text Clustering Algorithm

### 4.1. Improved Global K-Means Clustering Algorithm Analysis

In order to verify the real effect of clustering algorithm, the six data sets Iris, Wine, Soybean-small, Segmentation, Pima Indians Diabetes, and Pen digits are used for global clustering, fast global clustering, and improved clustering. By comparison of clustering time (*T*) sum of clustering error (*E*), we prove that the improved algorithm in this paper without seriously affecting the sum of squared of clustering errors. It greatly reduces the clustering time. Comparison of experimental results for the six sets of machine learning database data from UCl is shown in Table 1. Iris and Pen digits specifically refer to the data set of text big data in this paper.

From the above experimental results, compared with the other two algorithms, the improved algorithm obviously reduces the clustering time, without affecting the clustering error, right Soybean-small databases and databases greatly shorten the clustering time without seriously affecting the clustering errors. among Pen digits. It is particularly prominent in the big data sets. Thus, the present algorithm has a superior clustering performance.

In this paper, the improved global K-means clustering algorithm is tested by randomly generated artificial data sets with noise data to prove the anti-interference performance of the improved global K-means clustering algorithm against noise data. The randomly generated data are divided into three categories, each of which contains 120 two-dimensional samples, which conform to normal distribution. In class *i*, the mean value of abscissa *x* is *μ*_*x*_^*i*^, the mean value of ordinate is *μ*_*y*_^*i*^, and the standard deviation of class *i* is *σ*^*i*^. Among them, a certain number of noise points are added to the second class, and the standard deviation of the noise points is expressed as *σ*^*l*^. The effects of parameter category clustering for the three classes of randomly generated samples are shown in Table 2 and Figure 1. Figure 1 shows the clustering effect diagram of randomly generated three types of data, and its ordinate represents the time required for clustering the three types of data. The larger the value, the longer the time required.

The article "Research and Application of Clustering Algorithm for Text Big Data" was published in 2022. Journal: Comput Intell Neurosci.

These three sets of random data were tested using the above three algorithms, and the comparison of cluster time (*T*) and sum of cluster error (*E*) are shown in Table 3.

As can be seen from Table 3, these three algorithms have the same clustering effect on these three randomly generated data sets with noise points, but the improved algorithm in this paper has obvious advantages in clustering time, far superior to the other two kinds of algorithms. The steering results are shown in Figure 2. It can be seen from the table that the sum of squares of clustering errors of the three algorithms is the same, but the clustering time is gradually shortened, and the time required by this algorithm is the shortest, which also shows that this algorithm has obvious advantages in clustering time.

Visible from Figure 2, the global K-means algorithm, fast global K-means algorithm, and the improved global K-means algorithm in the three sets of randomly generated data sets with noise points has the same clustering effect, but this algorithm has obvious advantages in clustering time, far better than the global K-means algorithm and fast global K-means algorithm.

### 4.2. K-Means Original Algorithm and Improved Algorithm Analysis

In order to verify the effectiveness of the improved clustering algorithm, the Iris data set of the database was used for experimental test comparison. The comparative performance indexes are the accuracy and convergence rate (specifically the number of cycles of each test). First, the original and the improved algorithm were tested 10 random tests on the dataset, and the test metrics and accuracy comparisons are shown in Table 4 and Figure 3.

The original and the modified algorithms were subrandomly tested on the dataset, and the results on the loop number index are shown in Figure 4.

Figures 3 and 4 present the results of the experiment: the clustering accuracy of the original algorithm fluctuates between 79% and 89% and 89%, and the number of cycles fluctuates between the second times, while the accuracy of the improved algorithm is always 92%, and the number of cycles is always 3 times. The horizontal and vertical coordinates in Figure 4 represent the number of tests and the number of bad cycles, respectively. The number of bad cycles refers to the number of times it is necessary to classify these data in the process of substituting data into the algorithm for clustering. When the original algorithm is used for clustering in the figure, the number of times to follow the bad is uncertain, which shows that the algorithm is imperfect and the accuracy is unstable. The improved algorithm can be seen in the graph is very stable, which will greatly shorten the clustering time.

The article "Research and Application of Clustering Algorithm for Text Big Data" was published in 2022. Journal: Comput Intell Neurosci.

To verify the effectiveness of the improved algorithm in practical applications, the original K-means algorithm and the improved algorithm were tested 5 times, respectively, with the dataset, and the metrics randomly run 5 times are shown in Table 5.

The five tests are shown in Figure 5 in terms of the overall accuracy of the algorithm and in Figure 6 in terms of cycle times.

Figures 5 and 6 show the results of the experiment. The accuracy of the original algorithm fluctuates between times, and the cycle times fluctuate between the next times. Under the condition that the precision of the improved algorithm is unchanged, the number of cycles is unchanged, and the average time consumption is unchanged. Considering the experimental results, it is not difficult to see that the improved algorithm is better than the original algorithm in practice. At present, the automatic classification of text is widely used, such as Baidu news column display. For cluster analysis, category information is unknown and can automatically generate category information is not only critical for cluster mining count but also significant for subsequent data mining work.

## 5. Conclusion

Now, the data is explosive growth, and the data processing is particularly urgent. This paper studies big data processing, explains the concept and application of text big data, and introduces the processing method of text big data. This paper studies the clustering algorithm for text-oriented big data and analyzes the sample point similarity measure method and clustering algorithm. In this paper, the K-means algorithm is the main object to solve the adaptive clustering algorithm to optimize the initial clustering center of the clustering algorithm, in order to solve the problems such as failure to handle large-scale data sets, low clustering accuracy, and unstable clustering results. And, the original K-means algorithm of the original algorithm and improved algorithm, global K-means, and fast K-means algorithm, through a large number of real data comparison experiment, demonstrates the proposed new algorithm can solve the problems in the actual problem. Experimental results show that the algorithm is higher, and clustering results are more stable. In the era of big data, text data is exploding every day, and how to deal with text big data quickly and efficiently has become a difficult problem. The scientific significance of this paper lies in the research of clustering algorithm, bringing forth new ideas and putting forward new text data processing algorithm. It makes clustering algorithm more convenient and efficient to deal with practical problems.

The article "Research and Application of Clustering Algorithm for Text Big Data" was published in 2022. Journal: Comput Intell Neurosci.

## Figures and Tables

**Figure 1:** Cluster results diagram of the three categories.

**Figure 2:** Comparison of the cluster results for the randomly generated data.

**Figure 3:** Comparison plot of the accuracy of the original and improved algorithms for 10 random tests.

**Figure 4:** Comparison of the number of cycles of the original and improved algorithms.

**Figure 5:** Accuracy comparison of the original and improved algorithm randomly run 5 times.

**Figure 6:** Comparison of cycle number for five random runs of the original and improved algorithms.

**Table 1:** Comparison of the experimental results for several different clustering methods.

	The global K-means		Fast global K-means		The algorithm in this paper	
	*E*	*T* (*s*)	*E*	*T* (*s*)	*E*	*T* (*s*)
Iris	78.9408	0.438	78.9451	0.078	78.9451	0.031
Wine	2.3707 × 10^6^	0.765	2.707 × 10^6^	0.094	2.3707 × 10^6^	0.015
Soybean-small	96.3984	0.156	96.4702	0.047	96.4702	0
Segmentation	0.9398 × 10^6^	3.765	1.0076 × 10^6^	0.188	1.0198 × 10^6^	0.125
Pima Indians diabetes	5.1363 × 10^6^	3.625	5.1665 × 10^6^	0.109	5.1363 × 10^6^	0.047
Pen digits	9.9830 × 10^6^	186.391	1.0480 × 10^7^	6.844	1.0553 × 10^7^	0.953

**Table 2:** Randomly generated various parameters with the noise data.

	First kind	Second kind	The third class
Mean *μ*	*μ*_*x*_^1^=0	*μ*_*y*_^1^=0*μ*_*x*_^2^=6, *μ*_*y*_^2^=2	*μ*_*x*_^3^=6, *μ*_*y*_^3^=−1
Standard deviation *σ*	*σ* ^*i*^=1.5	*σ* ^2^=0.5, *σ*^*l*^=2	*σ* ^3^=0.5

**Table 3:** Comparison of the cluster results for the randomly generated data.

	*A*	*B*	*C*
*E* (×10^3^)	0.6363	0.6363	0.6363
*T* (*s*)	1.11	0.062	0.031

**Table 4:** The original algorithm and the improved algorithm are 10 random indicators.

Test serial number	The original algorithm		Improve the algorithm	
	Precision	Follow the bad times	Precision	Follow the bad times
1	84	10	93	3
2	83	5	92	3
3	89	7	90	3
4	82	4	92	3
5	85	13	92	3
6	84	3	92	3
7	83	10	89	3
8	79	4	85	3
9	89	5	92	3
10	89	9	92	3

**Table 5:** Five random runs of the original algorithm and the improved algorithm.

Test serial number	The original algorithm		Improve the algorithm	
	Precision	Follow the bad times	Precision	Follow the bad times
1	59	18	75	9
2	61	24	75	9
3	68	35	75	9
4	73	27	75	9
5	69	11	75	9

## Data Availability

The experimental data used to support the findings of this study are available from the corresponding author upon request.
